# Cantharidin Inhibits Proliferation of Liver Cancer by Inducing DNA Damage via KDM4A-Dependent Histone H3K36 Demethylation

**DOI:** 10.1155/2022/2197071

**Published:** 2022-07-11

**Authors:** Chao Wei, Xiangui Deng, Shudi Gao, Xuemei Wan, Jing Chen

**Affiliations:** ^1^Infectious Disease Department, Qijiang Hospital of the First Affiliated Hospital of Chongqing Medical University, Chongqing 401420, China; ^2^Infectious Disease Department, Wenlong Hospital of Qijiang, Chongqing 401420, China; ^3^Infectious Disease Department, Taiyuan Hospital of Traditional Chinese Medicine, Taiyuan 030009, Shanxi Province, China; ^4^Infectious Disease Department, Affiliated Hospital of Chengdu University of Traditional Chinese Medicine, Chengdu 610032, Sichuan Province, China

## Abstract

**Objective:**

To investigate the effect of cantharidin on DNA damage in hepatocellular carcinoma cells and its possible mechanism.

**Methods:**

Cell proliferation assay and terminal deoxynucleotidyl transferase-mediated dUTP nick end labeling (TUNEL) assay were used to analyze the effects of cantharidin on cell proliferation and apoptosis of hepatocellular carcinoma cells. The expression levels of DNA damage markers H2AX and P21 were analyzed by qRT-PCR. The expression of KDM4A and H3K36me3 was observed by western blot. The expression of KDM4A was regulated by siRNA or plasmid transfection. The effect of KDM4A on DNA damage induced by cantharidin in liver cancer was observed after overexpression and addiction of KDM4A.

**Results:**

Cantharidin can significantly inhibit the growth of hepatocellular carcinoma cells and induce apoptosis of hepatocellular carcinoma cells. Cantharidin enhances the chemotherapy sensitivity of liver cancer by targeting the upregulation of KDM4A and the regulation of DNA damage induced by H3K36me3. Overexpression of KDM4A enhances DNA damage induced by cantharidin in HCC. KDM4A silencing attenuated the damage of cantharidin to the DNA of HCC cells.

**Conclusion:**

Cantharidin can inhibit the growth and promote apoptosis of hepatocellular carcinoma cells. Meanwhile, cantharidin can induce DNA damage in HCC cells. Mechanism studies have shown that cantharidin induces DNA damage through the demethylation of KDM4A-dependent histone H3K36.

## 1. Introduction

Hepatocellular carcinoma (HCC), a solid tumor, is a malignant disease with a high frequency and mortality worldwide [1, 2]. Chemotherapy is the main treatment for advanced solid tumors [3–6].

Histone methylation is an important epigenetic modification [7, 8]. Lysine-specific demethylase 4A (KDM4A) specifically catalyzes the demethylation of histone lysine residues, thereby regulating the chromatin structure and gene transcription [9]. Studies have found that KDM4A is involved in the regulation of cell proliferation, differentiation, development, metabolism, and other important biological processes [10, 11]. Its abnormal function is also closely related to the occurrence and development of tumors and other diseases, becoming an important target for tumor therapy [12]. Histone methylation is one of the important epigenetic modifications, which plays an important role in many biological processes such as transcription activation and suppression, sex chromosome silencing, and DDR. Histone H3/H4 methylation mainly occurs at different leucine K sites (K4, K9, K27, K36, K79, and K20) [13]. The activation or suppression of chromosome transcription is related to methylation states such as monomethylation, demethylation, and trimethylation [14]. Histone methylation can regulate the function of DDR, thus affecting its tumor barrier role in DNA damage. H3K36me (histone H3 methylation at lysine 36) is the extension of the main influencing gene transcription process [15]. These histone modifications are abundant in the coding regions of transcription-activated genes. Studies on its role in DSB repair also showed that H3K36 methylation plays an important role in the NHEJ repair mode of DNA damage repair (DDR) [15].

Cantharidin can inhibit the protein synthesis of tumor cells, and then affect the synthesis of RNA and DNA and the progress of the cell cycle, promote the apoptosis of tumor cells, and inhibit the proliferation of tumor cells [16, 17]. It has been reported that cantharidin can induce apoptosis of HO-8910PM cells with high metastasis in human ovarian cancer [18, 19]. Cantharidin's promotion of tumor cell apoptosis is also related to the fact that cantharidin is a protein phosphatase inhibitor [20]. Cantharidin has a strong resistance to tumor cell invasion and metastasis. However, the detailed pharmacological mechanisms need to be further studied. In addition, whether cantharidin can induce DNA damage through KDM4A-dependent histone H3K36 demethylation has not been reported.

## 2. Methods

### 2.1. Cell Culture

HepG2 and SMMC-7721 cell lines were purchased from ATCC and cultured in a DMEM containing 10% fetal bovine serum, penicillin (100 U/mL), and streptomycin (100 g/mL). It was placed in a constant temperature incubator containing 5% CO_2_ at 37°C.

### 2.2. Cell Transfection

1 × 10^5^ SMMC-7721 and HepG2 cells were inoculated in 6-well plates with a 2 ml fresh complete medium. After overnight incubation, the medium was removed and a 2 ml medium containing siRNA KDM4A and a transfection reagent was added. After 24 h, the medium was removed and the 2 ml of fresh complete medium (DMEM + 10% FBS) was added to each well. After 48 h, transfection efficiency and subsequent experiments were tested.

### 2.3. TUNEL Analysis

The cells were prepared into cell suspension, which was respectively introduced into 6-well plates which had been added to the slides. The glass slide with good cells was immersed in 4% paraformaldehyde and fixed for 25 min. The cell slides were placed in 0.1% TritonX-100 prepared with PBS for 2 min. Treatment groups were mixed with a 50 *μ*L TdT + 450 *μ*L luciferase-labeled dUTP solution (the negative control group was added with 50 *μ*L luciferase-labeled dUTP solution). 50 *μ*l TUNEL reaction mixture was added and incubated at 37°C for 60 min away from the light. Each group was incubated with DAPI to avoid light for 5 min, and the samples were stained with nuclei. The tablets were sealed with a sealing solution, and then, the images were observed and collected under a fluorescence microscope. The number of TUNEL-positive cells was counted by the Image J software.

### 2.4. qRT-PCR

RNA was extracted and each sample was reverse-transcribed into cDNA according to a 20 *μ*l reaction system; reaction conditions were as follows: 42°C for 60 min and 95°C for 5 min. PCR was performed with cDNA as the template, and the quality of cDNA was checked by agarose gel electrophoresis. Then, according to the instructions of the real-time PCR kit, the reaction conditions were set as follows: 50°C for 2 min and 95°C for 10 min, (95°C, 30 s; 60°C, 30 s) × 40 cycles. The internal reference is GAPDH. Specific primer sequences are shown in Table 1. The expression levels of target genes were analyzed by RT-PCR and fluorescence quantitative PCR.

### 2.5. Histone Extraction

Cells were collected, followed by 1 mL/10^7^ cells, using Triton extraction buffer ((TEB: containing 0.5% TritonX-100 (V/V), 2 mmol/L phenylmethylsulfonyl fluoride (PMSF), 1% protease inhibitors, and phosphatase inhibitor in PBS) and the cells were resuspended. Under slow shaking, the cells were lysed on ice for 10 min and centrifuged at 2000 r/min for 10 min at 4°C. The supernatant was removed. The centrifugation was repeated again and the supernatant was discarded. 0.2 mol/L HCl was added and the cells were resuspended according to 1 mL/4 × 10^7^ cells. The histones were extracted at 4°C overnight. The supernatant was centrifuged and collected, that is, the histone extraction liquid.

### 2.6. Western Blot

Cells were seeded in 6-well plates at 5 × 10^5^ cells/well. After culturing for 24 h, different concentrations of cantharidin were added and incubated for 48 h. The total cell protein was extracted, and the concentration of the protein sample was determined by BCA and then mixed with 5 × protein loading buffer according to a loading amount of 30 *μ*g. It was boiled in water for 5 min to denature it. The samples for SDS-PAGE were taken. The target protein was transferred on the separation gel to the PVDF membrane by all-wet electroporation. 5% skimmed milk powder was blocked for 1 h. After complete blocking, the primary antibody (1: 1000) was added and incubated at 4°C overnight. The secondary antibody (1: 1000) was added and incubated at room temperature for 2 h. Chemiluminescence detection of the target band, and observation and analysis of the gel imaging system and photographing were performed. The amount of target protein was calculated by the ratio of the absorbance values of the target protein and the internal reference protein.

### 2.7. Cell Proliferation Assay

Cells in the logarithmic growth phase were seeded at 5 × 10^3^/well in 96-well plates. 200 *μ*l per well, and drug treatment was added after 24 hours when the cells had grown to a density of about 50%. Cells were collected after 48 h for CCK-8 experiments. The blank group, negative control group, and drug-treated group without the cells and only the medium were set up with 3 replicate wells in each group following the instructions of the CCK-8 kit. The absorbance value (A value) at 450 nm wavelength of each well was read with a microplate reader.

### 2.8. Statistical Analysis

The above experiments were repeated three times, and the experimental results were expressed as mean ± standard deviation (mean ± standard deviation). SPSS 17.0 software was used for statistical analysis. The *t* test was used for the comparison between the two groups, the data between multiple groups were analyzed by one-way analysis of variance, and pairwise comparison between the groups was performed by the LSD *t* test.

## 3. Results

### 3.1. Effects of Cantharidin on the Viability and Apoptosis of Hepatoma HepG2 and SMMC-7721 Cells

The growth of HepG2 and SMMC-7721 cells was significantly inhibited by cantharidin stimulation for 48 h. The growth inhibition rates of HepG2 and SMMC-7721 cells increased with the increase of cantharidin concentration (Figures 1(a) and 1(b)). Apoptosis was further detected by the TUNEL assay. The results showed that the apoptosis rate of SMMC-7721 cells increased after cantharidin treatment (Figures 1(c) and 1(d)).

### 3.2. Cantharidin Induces DNA Damage and Enhances Chemotherapy Sensitivity of Liver Cancer

HepG2 and SMMC-7721 cells were treated with cantharidin (10 *μ*M) for 48 h. After cytoplasmic nucleus isolation, the expression of DNA damage markers H2AX and P21 in the nucleus was detected by qRT-PCR. The results showed that H2AX and P21 expressions increased after cantharidin stimulation (Figures 2(a) and 2(b)). These results indicated that cantharidin treatment could increase DNA damage in cells. Subsequently, we conducted cell proliferation experiments to verify whether cantharidin can increase the antitumor effect of HCC chemotherapy drugs. Results showed that the cell viability of HepG2 and SMMC-7721 was significantly decreased in 20 *μ*M sorafenib combined with cantharidin (10 *μ*M) compared to the group given sorafenib alone (Figures 2(c) and 2(d)).

### 3.3. Cantharidin Upregulated the Expression of KDM4A

The expression of KDM4A mRNA in HepG2 and SMMC-7721 hepatoma cell lines treated with cantharidin was detected by qRT-PCR. The results showed that the expression of KDM4A in HepG2 and SMMC-7721 cells was significantly increased after cantharidin stimulation (Figure 3(a)). The expression of KDM4A and histone methyltransferase H3K36me3 was detected by western blotting. The results showed that the KDM4A expression was upregulated and the H3K36me3 expression was downregulated in HepG2 and SMMC-7721 cells after cantharidin treatment (Figure 3(b)). These results suggest that cantharidin may increase DNA damage by affecting H3K36me3.

### 3.4. Overexpression of KDM4A Enhances DNA Damage Induced by Cantharidin in Liver Cancer

The expression of KDM4A in HepG2 and SMMC-7721 cells with KDM4A overexpression (KDM4A-OE) was detected by qRT-PCR. Experimental results showed that the expression level of KDM4A was upregulated in the overexpression group (Figure 4(a)). Western blot was used to detect the expression of KDM4A and H3K36me3 in normal and KDM4A-overexpressed liver cancer cells and cantharidin-treated groups. The results showed that compared with the control group, the expression level of KDM4A was upregulated in both cantharidin stimulation and KDM4A overexpression groups. The expression level of the KDM4A + cantharidin treatment group was the highest. Compared with the control group, both cantharidin stimulation and KDM4A overexpression could inhibit the expression of H3K36me3. Meanwhile, the expression level of H3K36me3 in the treatment group with simultaneous overexpression of KDM4A + cantharidin was the lowest (Figure 4(b)). The expression levels of H2AX and P21 were detected after different treatments, and the DNA damage of HCC cells was analyzed. The results showed that after cantharidin + overexpression KDM4A combined treatment, H2AX and P21 had the highest expression (Figures 4(c) and 4(d)). Cell activity detection experiments also showed that the cell activity was the lowest after cantharidin + KDM4A overexpression combined treatment (Figure 4(e)). These results indicate that overexpression of KDM4A enhances DNA damage induced by cantharidin in liver cancer.

### 3.5. KDM4A Silencing Can Weaken the Damage of Cantharidin to the DNA of HCC Cells

The mRNA levels of KDM4A in HepG2 and SMMC-7721 cells were detected by qRT-PCR. The results showed that siRNA could significantly reduce the expression level of KDM4A (Figure 5(a)). Western blot results showed that compared with the cantharidin treatment group, siRNA KDM4A + cantharidin treatment decreased the KDM4A expression, while the H3K36me3 expression was upregulated (Figure 5(b)). Results of H2AX and P21 expression detection showed that H2AX and P21 expression levels decreased in the siRNA KDM4A + cantharidin treatment group compared to Figures 5(c) and 5(d). Cell activity detection experiments also showed that compared with the cantharidin treatment group, the cell activity increased after cantharidin + siRNA KDM4A combined treatment (Figure 5(e)). These results suggest that KDM4A silencing can attenuate the damage of cantharidin to the DNA of HCC cells.

## 4. Discussion

Liver cancer has a very negative impact on people's health and life, and so far, there is no effective treatment [21, 22]. Changes in the cell's internal and external environment often lead to DNA molecular damage and structural changes. DNA double-strand break (DSB) is one of the most serious manifestations of DNA damage [23]. On the other hand, the current treatment of tumors is often carried out by destroying the DNA in tumor cells [24, 25].

As a key epigenetic enzyme regulating gene expression, abnormal activity of KDM4A is associated with the occurrence of a variety of tumors [26]. KDM4A overexpression can significantly block the regulation of miR-526b on cell growth and invasion, thus promoting the growth of gastric cancer cells [27]. Neault et al. [28] found that mir-137 targets KDM4A mRNA and activates p53 in pancreatic cancer cells, inhibiting cell proliferation. In the treatment of pancreatic cancer, fisetin can induce the expression of RFXAP (regulatory factor X-associated protein), which leads to the upregulation of the KDM4A expression and the downregulation of H3K36 methylation, thus inhibiting the DNA damage repair pathway [29]. KDM4A is the target gene of RFX5 (regulatory factor X-5) in hepatocellular carcinoma cells. The Rfx5-kdm4a pathway promotes the process of the cell cycle from the G0/G1 phase to the S phase and inhibits apoptosis [30]. Due to the important role of KDM4A in tumor genesis and treatment, the study of KDM4A inhibitors is particularly important. Targeting KDM4A has become a hot topic in the treatment of tumors. The KDM4A inhibitor JIB-04 can restore the level of H3K36me3 and the sensitivity of tumor cells to cytarabine [31]. JIB-04 is a small molecule inhibitor that can destroy the binding between KDM4A and oxygen molecules [32]. In this study, the antitumor effect of cantharidin and its increasing antitumor effect of sorafenib are related to the inhibition of KDM4A.

Histone methylation may play an important regulatory role in DNA damage response. The subsequent discovery of histone demethylase proved the reversibility of this modification process. Histone H2AX is a biomarker of DNA double-strand break in vivo [33]. It plays an important role in DNA damage signal transduction and the recruitment of repair proteins. H2AX is also closely related to genome stability, cell cycle, and apoptosis [34]. H2AX is closely related to the occurrence and development of tumors [35, 36]. By detecting the changes of DNA damage markers H2AX and P21, the occurrence of DSBs in HCC cells under different time and concentration gradient conditions was observed. The expression levels of H2AX and P21 increased with cantharidin stimulation. This is a manifestation of DNA damage caused by cantharidin.

Due to KDM4A's versatility, this study further investigated the role of the KDM4A gene in DNA damage of tumor cells induced by chemotherapeutic drugs. The effect of KDM4A gene silencing on cantharidin-induced DNA damage in hepatocellular carcinoma cells was observed by transfection of the KDM4A-OE overexpressed plasmid. It was confirmed that the DNA damage of hepatoma cells transfected with the KDM4A-OE interfering plasmid was increased compared with the control cells under the treatment of cantharidin (10 *μ*M). The reason may be that the expression of the KDM4A gene is upregulation; therefore, DNA damage repair is obstructed and the cells cannot repair broken DNA in time, thus promoting DNA damage induced by cantharidin.

This study found that cantharidin can inhibit liver cancer by promoting DNA damage. The promotion of DNA damage is achieved by acting on KDM4A. In this study, we found that cantharidin can regulate epigenetic effects of tumors and then play an antitumor effect. The research on the pharmacological action of antitumor drugs has a reference significance.

## 5. Conclusion

In conclusion, cantharidin can reduce the survival rate of HCC cells and promote the occurrence of DNA damage. Transfection of the KDM4A overexpressed plasmid can upregulate the expression of KDM4A and promote DNA damage of hepatoma cells induced by cantharidin. In addition, cantharidin induces DNA damage and enhances chemotherapy sensitivity of liver cancer. Mechanism studies suggest that cantharidin induces DNA damage through KDM4A-dependent demethylation of histone H3K36. The results of this study provide a new reference for the combined application of cantharidin with chemotherapy drugs.

## Figures and Tables

**Figure 1:** The effect of cantharidin on the in vitro activity of hepatocellular carcinoma. (a) CCK-8 detection of HepG2 cells. Cells were treated with cantharidin (10 *μ*M) for 48 h. Absorbance was measured at 450 nm. (b) CCK-8 detection of SMMC-7721 cells. Cells were treated with cantharidin (10 *μ*M) for 48 h. Absorbance was measured at 450 nm. (c) Apoptosis of cells after treatment. SMMC-7721 cells were treated with cantharidin (10 *μ*M) for 48 h and analyzed by the TUNEL assay. (d) Apoptosis statistical analysis results.  ^*∗*^ ^*∗*^*p* < 0.01.

**Figure 2:** Cantharidin induces DNA damage and enhances chemosensitivity in liver cancer. (a) The expression of the DNA damage marker H2AX in the nucleus was detected by qRT-PCR after cytoplasmic nucleus isolation. HepG2 and SMMC-7721 cells were treated with cantharidin (10 *μ*M) for 48 h, respectively. (b) The expression of the DNA damage marker p21 in the nucleus was detected by qRT-PCR after separation of the cytoplasm and the nucleus. HepG2 and SMMC-7721 cells were treated with cantharidin (10 *μ*M) for 48 h, respectively. (c) Sorafenib (20 *μ*M) and cantharidin (10 *μ*M) combined treatment significantly decreased the viability of HepG2 cells. (d) The viability of SMMC-7721 cells was significantly decreased after sorafenib (20 *μ*M) and cantharidin (10 *μ*M) were combined.  ^*∗*^*p* < 0.05,  ^*∗*^ ^*∗*^*p* < 0.01.

**Figure 3:** Cantharidin upregulated the KDM4A expression. (a) The expression of KDM4A mRNA in liver cancer cell lines HepG2 and SMMC-7721 after cantharidin treatment was detected by qRT-PCR. (b) Western blot detection of KDM4A and H3K36me3 expressions in hepatoma cells treated with cantharidin. Data are presented as mean ± SD (*n* = 3),  ^*∗*^ ^*∗*^*p* < 0.01.

**Figure 4:** Overexpression of KDM4A enhances cantharidin-induced DNA damage in liver cancer. (a) qRT-PCR of KDM4A in the control and KDM4A-overexpressing (KDM4A-oe) HepG2 and SMMC-7721 cells. (b) The expression of KDM4A and H3K36me3 in the normal and KDM4A-overexpressed hepatoma cells and in cantharidin-treated group. (c) The expression of H2AX was detected after different treatments, and the DNA damage of liver cancer cells was analyzed. KDM4A-HepG2 cells were treated with cantharidin (10 *μ*M) for 48 h. (d) The expression of p21 was detected after different treatments, and the DNA damage of liver cancer cells was analyzed. KDM4A-HepG2 cells were treated with cantharidin (10 *μ*M) for 48 h. (e) Detection of CCK-8 in HepG2 cells overexpressing KDM4A. Cells were treated with cantharidin (10 *μ*M) for 48 h.  ^*∗*^*p* < 0.05,  ^*∗*^ ^*∗*^*p* < 0.01.

**Figure 5:** KDM4A silencing attenuates cantharidin-induced DNA damage in hepatoma cells. (a) KDM4A mRNA levels in the control and KDM4A silenced (siRNA) HepG2 were detected by qRT-PCR. (b) Western blot detection of KDM4A and H3K36me3 expression changes. KDM4Ai-HepG2 cells were treated with cantharidin (10 *μ*M) for 48 h. (c) The expression of H2AX was detected after different treatments, and the DNA damage of liver cancer cells was analyzed. KDM4Ai-HepG2 cells were treated with cantharidin (10 *μ*M) for 48 h. (d) The expression of p21 was detected after different treatments, and the DNA damage of liver cancer cells was analyzed. Cells were treated with cantharidin (10 *μ*M) for 48 h. (e) CCK-8 detection of HepG2 cells with siRNA KDM4A. Cells were treated with cantharidin (10 *μ*M) for 48 h.  ^*∗*^*p* < 0.05,  ^*∗*^ ^*∗*^*p* < 0.01.

**Table 1:** Primer sequence.

Genes	Sequences (5′-3′)
H2AX	F: CGGGCGTCTGTTCTAGTGTT
	R: GGTGTAC ACGGCCCACTG

p21	F: TGTCCGTCAGAACCCATGC
	R: AAAGTCGAAGTTCCATCGCTC

KDM4A	F: GCCGCTAGAAGTTTCAGTGAG
	R: GCGTCCCTTGGACTTCTTATT

GAPDH	F: GTATAATGAGAAGCCAGACCAT
	R: ACAGCTTCTCAAGTCT

## Data Availability

The data used to support the findings of this study are available from the corresponding author upon request.
